The article "Identifying Coronary Artery Lesions by Feature Analysis of Radial Pulse Wave: A Case-Control Study" was published in 2021. Journal: Biomed Res Int.

# Identifying Coronary Artery Lesions by Feature Analysis of Radial Pulse Wave: A Case-Control Study

**DOI:** 10.1155/2021/5047501

**Published:** 2021-12-30

**Authors:** Chun-ke Zhang, Lu Liu, Wen-jie Wu, Yi-qin Wang, Hai-xia Yan, Rui Guo, Jian-jun Yan

**Affiliations:** ^1^Department of Basic Medical Science, Shanghai Key Laboratory of Health Identification and Assessment, Shanghai University of Traditional Chinese Medicine, 1200 Cailun Road, Pudong New District, Shanghai 201203, China; ^2^Institute of Intelligent Perception and Diagnosis, School of Mechanical and Power Engineering, East China University of Science and Technology, 130 Meilong Road, Xuhui District, Shanghai 200237, China

## Abstract

**Background:**

Cardiovascular diseases have been always the most common cause of morbidity and mortality worldwide. Health monitoring of high-risk and suspected patients is essential. Currently, invasive coronary angiography is still the most direct and accurate method of determining the severity of coronary artery lesions, but it may not be the optimal clinical choice for suspected patients who had clinical symptoms of coronary heart disease (CHD) such as chest pain but no coronary artery lesion. Modern medical research indicates that radial pulse waves contain substantial pathophysiologic information about the cardiovascular and circulation systems; therefore, analysis of these waves could be a noninvasive technique for assessing cardiovascular disease.

**Objective:**

The objective of this study was to analyze the radial pulse wave to construct models for assessing the extent of coronary artery lesions based on pulse features and investigate the latent value of noninvasive detection technology based on pulse wave in the evaluation of cardiovascular disease, so as to promote the development of wearable devices and mobile medicine.

**Method:**

This study included 529 patients suspected of CHD who had undergone coronary angiography. Patients were sorted into a control group with no lesions, a 1 or 2 lesion group, and a multiple (3 or more) lesion group as determined by coronary angiography. The linear time-domain features and the nonlinear multiscale entropy features of their radial pulse wave signals were compared, and these features were used to construct models for identifying the range of coronary artery lesions using the *k*-nearest neighbor (KNN), decision tree (DT), and random forest (RF) machine learning algorithms. The average precision of these algorithms was then compared.

**Results:**

(1) Compared with the control group, the group with 1 or 2 lesions had increases in their radial pulse wave time-domain features H2/H1, H3/H1, and W2 (*P* < 0.05), whereas the group with multiple lesions had decreases in MSE1, MSE2, MSE3, MSE4, and MSE5 (*P* < 0.05). (2) Compared with the 1 or 2 lesion group, the multiple lesion group had increases in T1/T (*P* < 0.05) and decreases in T and W1 (*P* < 0.05). (3) The RF model for identifying numbers of coronary artery lesions had a higher average precision than the models built with KNN or DT. Furthermore, average precision of the model was highest (80.98%) if both time-domain features and multiscale entropy features of radial pulse signals were used to construct the model.

The article "Identifying Coronary Artery Lesions by Feature Analysis of Radial Pulse Wave: A Case-Control Study" was published in 2021. Journal: Biomed Res Int.

**Conclusion:**

Pulse wave signal can identify the range of coronary artery lesions with acceptable accuracy; this result is promising valuable for assessing the severity of coronary artery lesions. The technique could be used to development of mobile medical treatments or remote home monitoring systems for patients suspected or those at high risk of coronary atherosclerotic heart disease.

## 1. Introduction

Cardiovascular diseases (CVD) are the highest cause of mortality and morbidity all over the world [1]. In the United States, one person dies from CVD every 33 seconds, and 70% of those deaths are from coronary heart disease (CHD). In China, the number of patients with CHD rose to 11 million in 2019, and the CHD mortality rate continues to rise [2]. CHD is now a significant and global public health problem that has attracted the attention of medical researchers worldwide.

Coronary angiography can determine the position and number of coronary artery lesions to assess the severity of a patient's condition [3]. However, research has demonstrated [4–6] that, among patients with suspected CHD who have symptoms of chest pain, coronary angiography did not identify CHD in numerous cases. The prevalence of coronary artery stenosis was more likely to be overestimated among elderly patients. Furthermore, coronary angiography is an invasive operation and is correlated with death, myocardial infarctions, and other severe complications such as vascular injury or hematoma [7, 8]. Therefore, noninvasive methods of detecting the severity of coronary artery lesions in patients with suspected CHD have received substantial recent attention.

A pulse wave is excited by cardiac ejection. The fluctuation of the radial artery pulse wave corresponds to the events constituting the cardiac cycle [9]. The pressure pulse wave can be measured at the radial artery, because the radial artery is shallow and its diameter is relatively thick, which is easy to touch and is not easily disturbed by subcutaneous tissue, fat, and other factors. Modern research has indicated that features of the pressure pulse wave in the radial artery can reveal arterial stiffness and indicate cardiovascular function [10, 11]. It is recognized that atherosclerosis affects blood vessels throughout the body; coronary atherosclerosis has the same pathological mechanism as large- and medium-sized elastic arteries. Therefore, arteriosclerosis indicators can be used to assess the degree of coronary atherosclerosis [12]; thus, assessing the extent of coronary arterial lesions based on pulse wave analysis techniques is feasible.

The article "Identifying Coronary Artery Lesions by Feature Analysis of Radial Pulse Wave: A Case-Control Study" was published in 2021. Journal: Biomed Res Int.

The time-domain method, a most frequently used method for pulse signal analysis, is able to extract amplitudes and phases of a cardiac cycle of pulse signal. These amplitudes and phases have specific pathophysiological implication reflecting the cardiovascular status. Qi et al. [10] incorporated radial pulse wave time-domain feature H3/H1 reflecting peripheral vascular resistance and arterial stiffness into a hypertension risk prediction model and compared it with the model using Ba-PWV. The results revealed that the model using time-domain H3/H1 of pulse signal as a predicting factor had higher accuracy in predicting hypertension risk. The human body is a complex system with numerous coupling dynamics expressed in nonlinear forms. Human physiological signals, such as pulse wave signals, also have nonlinear features [13]. Nonlinear analytical methods have become the primary method of analyzing biomedical signals. Wang et al. [14] used approximate entropy to analyze the pulse signals of patients with cardiovascular diseases. They observed that, compared with the pulse signals of healthy individuals, the pulse signals of patients with cardiovascular diseases had lower entropy and fewer irregularities. Yan et al. [15] used Lyapunov indicators to compare the pulse signals of patients with CHD and healthy individuals and found differences that demonstrated this nonlinear analysis can be used to detect CHD in patients. Therefore, in this paper, linear and nonlinear analytical methods were employed to extract pulse features for revealing the cardiovascular information hidden in pulse wave from different perspectives.

Effective risk stratification can lower patient incidence of disease and lower the possibility of the patient undergoing invasive diagnostic procedures. However, precise risk stratification prediction models require substantial amounts of data and follow-up research to build, and the rapid development of artificial intelligence has enabled machine learning algorithms to convert small samples of clinical data into more precise prediction models [16]. These models can be used in long-term disease tracking, management, and feedback in mobile medical devices, enabling new options for the early diagnosis of diseases and the management of chronic diseases [17]. Research in applying machine learning methods has yielded some achievements in the establishment of cardiovascular disease models based on radial pulse wave signals [18, 19].

The article "Identifying Coronary Artery Lesions by Feature Analysis of Radial Pulse Wave: A Case-Control Study" was published in 2021. Journal: Biomed Res Int.

This study involves obtaining pulse wave signals from the arterial artery by using noninvasive pulse detection equipment, extracting the time-domain features and the multiscale entropy features, and finally grouping patients by number of coronary artery lesions in accordance with coronary angiography results to identify differences in time-domain features and multiscale entropy features of pulse wave. Models for assessing the severity of coronary artery lesions were also built on the basis of different datasets and multiple machine learning algorithms to investigate the latent value of radial pulse wave in assessing the extent of coronary artery lesions as well as the potential of pulse waves for individual medical monitoring of patients.

## 2. Methods

### 2.1. Research Participants

The research participants were 529 patients previously suspected to have CHD and who underwent coronary angiography between December 2019 and December 2020 from departments of cardiology in two hospitals in Shanghai, including Yueyang Hospital of Integrated Traditional Chinese and Western Medicine, and Shuguang Hospital, which are affiliated to Shanghai University of Traditional Chinese Medicine.

Based on the coronary angiographs, patients with lesions of less than 50% diameter stenosis were assigned to the control group (Group 1), whereas patients with lesions of greater than 50% diameter stenosis were further sorted by the number of coronary artery lesions, specifically those with 1 or 2 lesions (Group 2) and multiple (3 or more) lesions (Group 3) [20].

Participants were excluded if they had chest pains caused by other heart diseases, severe neurosis, with atrial fibrillation/flutter or aortic valve stenosis, a history of percutaneous coronary intervention surgeries or coronary artery bypass surgery, or incomplete clinical medical records.

The Medical Ethics Committee of the Yueyang Hospital of Integrated Traditional Chinese and Western Medicine affiliated to Shanghai University of Traditional Chinese Medicine approved the study (Approval number: 2020-175), and written informed consent was obtained from all included subjects according to the Declaration of Helsinki.

### 2.2. Pulse Collection

The patients' pulse waves were collected using a ZBOX-I pulse detection equipment (product by: Shanghai Asia & Pacific Computer Information System Co., Ltd., Shanghai, China). This pulse detection equipment was mentioned in our previous study [21] and has a wide range of applications in the research of cardiovascular diseases [22–24]. Each subject was instructed to relax for more than 5 min before pulse wave was recorded. The pulse wave recordings of all subjects were measured in styloid process of the radius where the radial artery pulsates of the left hand, the best position to feel the pulse, and recorded for 60 sec at a sample rate of 720 Hz.

The article "Identifying Coronary Artery Lesions by Feature Analysis of Radial Pulse Wave: A Case-Control Study" was published in 2021. Journal: Biomed Res Int.

### 2.3. Method of Pulse Feature Extraction

In this study, the features of the radial pulse wave signals were extracted using time-domain analysis and multiscale entropy analysis.

#### 2.3.1. Time-Domain Analysis

The time-domain analysis is a method that mainly quantifies the characteristic points of the pulse waveform in a single cardiac cycle. As shown in Figure 1, in a cardiac cycle of pulse waveform, the peak point and valley point of the waveform including the starting point and ending point are feature points with physiological significance. They are as follows: H1: the height of percussion wave (main wave), H2: the height of main wave gorge, H3: the height of tidal wave, H4: the height of dicrotic notch, H5: the height of dicrotic wave, T1: main wave phase, T2: main wave gorge phase, T3: tidal wave phase, T4: the dicrotic notch phase, T5: the dicrotic notch phase, T: pulse cycle, w1: the width of main wave in its 1/3 height position, and W2: the width of main wave in its 1/3 height position.

The classical time-domain features were extracted in this study, which were H2/H1, H3/H1, H4/H1, H5/H1, T1/T, T1/T4, T, W1, and W2. Their physiological significances are presented in Table 1.

#### 2.3.2. Multiscale Entropy Analysis

Multiscale entropy analysis is a nonlinear method. It was proposed by Costa et al. to evaluate the complexity of time series by taking into account the multiple time scales in physical systems, and soon, these approaches have been used in biosignals to estimate the degree of randomness or regularity in physiological processes [25, 26]. Multiscale entropy analysis can determine low self-similarity across scales and requires a coarse-grained procedure of the signals and the entropy computation for the original signal and for the coarse-grained time series (Figure 2). The method is as follows:

(1) $$\begin{array}{c} y_{j}^{\left(s\right)}=\frac{1}{s}\overset{js}{\underset{i=\left(j-1\right)s+1}{\sum }}u_{i},1\leq j\leq \frac{N}{s}. \end{array}$$

Here, *s* denotes the scale factor, *u* is the initial signal to be tested, and *y* is the coarse-grained signal. If the scale factor is 1, *y* is equal to *u*. In this study, 5 was set as the maximum scale factor. We averaged data for each scale factor (*m* = 1, ⋯, 5), and we used the MSE method, as originally proposed [21] for calculation of MSEi (*i* = 1, ⋯, 5).

The article "Identifying Coronary Artery Lesions by Feature Analysis of Radial Pulse Wave: A Case-Control Study" was published in 2021. Journal: Biomed Res Int.

MSEi (*i* = 1, ⋯, 5) were used to analyze the complexity of the radial pulse wave signal at 5 scales.

### 2.4. Statistical Analysis

Analysis was performed using statistical software SPSS 25.0 (IBM, Armonk, NY) to compare the baseline features and radial pulse wave features of patients with different groups.

Continuous variables were compared using the Wilcoxon-Mann-Whitney nonparametric test, and categorical variables were compared using the chi-squared test. The continuous variables were expressed as median values and quartile ([M (Q1, Q3)]), and the categorical variables were expressed in percentages. All reported *P* values were 2-tailed, and those <0.05 were considered statistically significant.

### 2.5. Machine Learning Methods

The 3 machine algorithms—*k*-nearest neighbors (KNN), decision tree (DT), and random forest (RF)—were used to build models. KNN is a simple method of machine learning, which could classify unlabeled observations by assigning them to the class of the most similar labeled examples [27]. DT is a method of classification and regression. In the DT, the tree models are composed of nodes and directed edges, and optimal classifications are achieved through learning processes that involve recursive feature selection, DT generation, and pruning [28]. RF uses a large series of decision trees with low reciprocal correlation and randomly selected features using the method of bagging to obtain more precise and stable classifications and predictions [29].

## 3. Results

### 3.1. Baseline Information of Patients with Different Numbers of Coronary Artery Lesions

The baseline characteristics of 529 participants is shown in Table 2.

### 3.2. Comparison of Time-Domain Features

The comparison of time-domain features between groups with different numbers of coronary artery lesions in the total studied population is shown in Table 3. Compared with Group 1, Group 2 had increases in time-domain features H2/H1, H3/H1, and W2 (*P* < 0.05); compared with group 2, Group 3 had increases in T1/T (*P* < 0.05) and decreases in T and W1 (*P* < 0.05).

### 3.3. Comparison of Multiscale Entropy Features

The comparison of multiscale entropy features between the three groups is shown in Table 4. Table 4 indicates that, compared with Group 1, Group 3 had lower MSE1, MSE2, MSE3, MSE4, and MSE5 (*P* < 0.05).

### 3.4. Models Assessing Different Extents of Coronary Artery Lesions Based on Pulse Wave

By using the demographics of the patients (*n* = 529) suspected of having CHD—age, sex, and BMI–as baseline dataset, their pulse wave time-domain features and MSE features were used to form 3 sets of feature dataset. These datasets were Dataset 1 (baseline dataset and time-domain features), Dataset 2 (baseline dataset and MSE features), and Dataset 3 (baseline dataset, time-domain features, and MSE features). The performance of each model was then assessed using its average precision. Models for identifying different numbers of coronary artery lesions were built, respectively, using KNN, DT, and RF machine learning algorithms for each dataset, as presented in Table 5.

The article "Identifying Coronary Artery Lesions by Feature Analysis of Radial Pulse Wave: A Case-Control Study" was published in 2021. Journal: Biomed Res Int.

Table 5 indicates that, compared with KNN and DT, the RF-based models had higher average precisions (74.25% for Dataset 1, 80.15% for Dataset 2, and 80.98% for Dataset 3) than the KNN-based model and DT-based model. For another, compared with Dataset 1 and Dataset 2, the recognition precision of Group 1 and Group 3 by the RF-based model with Dataset 3 was the highest (89.16% for Group 1 and 86.65% for Group 2), respectively.

## 4. Discussion

CHD's leading risk factors include age, sex, diabetes, hypertension, and hyperlipidemia [30–34]. These risk factors cause lipids to be continuously deposited along the inner walls of blood vessels, forming plaque. Atherosclerotic plaque on the inner membrane of the coronary arteries, affected by vasoconstriction, manifests as crescent shapes and is heavier on the myocardial side [35]. On the side without plaque, the smooth muscle and elastic fibers within the arterial wall can still maintain some constriction and elasticity, which may have a compensatory effect on the blood supply of the coronary arteries. Therefore, for coronary arteries with few lesions, blockages in the coronary arteries result in lower arterial compliance and increased peripheral resistance. If the number of lesions in the coronary arteries increases, long-term and chronic blockages result in weakening of the compensatory ability, reduced myocardial perfusion reserve, and significantly lowered left ventricular function; these lead to higher mortality [36, 37].

In this study, the average age of the participants in Group 3 was higher than that of the participants in Group 1(*P* < 0.05). Furthermore, group 2 and group 3 with coronary artery lesions had fewer women and more men than the control group (*P* < 0.05). These sex differences were more evident with greater coronary artery lesions, and it was consistent with the existing finding that the gender difference was also found in coronary calcification [38]. This result may be partly due to the protective effects of estrogen for atherosclerosis [39]. Complications such as hypertension and diabetes were also more common in groups with more coronary artery lesions (Groups 2 and 3) than those in the control group (*P* < 0.05). Hypertension and diabetes are both independent risk factors for CHD and exacerbate atherosclerotic lesions. Prolonged hypertension and diabetes aggravated CHD and increased its incidence. Participants in Group 2 had lower systolic pressure than the control group (*P* < 0.05). In fact, lower systolic pressure is associated with poor outcomes of cardiovascular events [40].

The article "Identifying Coronary Artery Lesions by Feature Analysis of Radial Pulse Wave: A Case-Control Study" was published in 2021. Journal: Biomed Res Int.

CHD occurs due to the combined effects of multiple risk factors. Pulse waves include cardiovascular information about cardiac ejection activity and the propagation of the pulse along the vascular tree, and changes in of structure and function of the coronary arteries inevitably lead to corresponding changes of the pulse wave. Therefore, time-domain features and MSE features of pulse wave could indicate those changes in CHD.

Increases in H2/H1 and H3/H1 indicate that, as the number of lesions in the coronary arteries increases, aortic compliance decreases and peripheral resistance increases. An increase in W2 indicates that high arterial pressure has been maintained for a prolonged period of time. Compared with Group 2, Group 3 with a greater number of lesions in the coronary arteries had higher T1/T and lower T and W1 (*P* < 0.05). Those outcomes indicated that Group 3 has significantly weakened myocardial contractility, resulting in limited cardiac ejection capacity and insufficient circulating blood volume in the arteries, and the duration of intravascular hypertension in arteries is relatively shortened. The heart rate increases to compensate for this phenomenon and increase the total cardiac output.

MSE is a method of measuring the complexity of time series. Entropy-based measurements are widely used to quantify the complexity of various biomedical time-series datasets [41]. The results of this study revealed that, compared with Group 1, Group 3 had lower MSE1, MSE2, MSE3, MSE4, and MSE5 (*P* < 0.05). Greater entropy values indicate that the signals generated by the system are more random and irregular, indicating that the system has lower complexity. Furthermore, reduction of complexity is a common feature of pathodynamics [42]. Therefore, MSE features reflect that, as the number of coronary artery lesions increases, the regulatory ability of the cardiovascular system worsens. As demonstrated in other studies, compared with healthy people, people with cardiovascular diseases typically have reduced entropy values, and changes in the entropy value indicate changes in the cardiovascular regulatory system mediated by the autonomic nervous system [25, 41, 43]. The complexity of cardiovascular systems of various pathological states can be differentiated using pulse wave MSE features.

The article "Identifying Coronary Artery Lesions by Feature Analysis of Radial Pulse Wave: A Case-Control Study" was published in 2021. Journal: Biomed Res Int.

Following technological advances, computing tools for processing diagnostic information have been increasingly used to study the biomedical information of patients with cardiovascular diseases [44]. Existing research [36] has demonstrated that machine learning algorithms can produce accurate results when sorting epidemiological data. The random forest, a key data mining method in machine learning field that depends on a computer to learn all the complicated and nonlinear interactions among variables through minimization of errors between observed and predicted outcomes, can achieve a higher accuracy in the disease prediction by using bootstrap aggregation and randomization of predictors [29]. Besides, RF models are less prone to overfitting. In this study, the model built using RF algorithms had a higher average precision than the models built with KNN or DT algorithms. Furthermore, the model average precision was highest when both the time-domain features and multiscale entropy features were included.

Due to the high prevalence of CHD and the serious harm it causes, the aim of this study is to assess the extent of coronary artery disease through a noninvasive, traceable, out-of-hospital method to help people at risk and patients with CHD know their coronary condition and make timely adjustments to their potentially modifiable risk factors. Over the past few decades, wearable devices that monitor physiological signals have been increasingly used in diagnostics and treatments and have played an important role in medicine and health care. This study may be a reference for the development of wearable devices that can detect cardiovascular lesions.

## 5. Conclusion

Radial pulse signals can be used as an indicator of the extent of coronary artery lesions. Models for assessing coronary artery lesions based on pulse detection techniques are useful for determining the severity of coronary artery lesions. Therefore, these models could be used to develop remote health monitoring based on noninvasive and wearable radial pulse wave signals and combined with actuators and modern communication and information technology system for monitoring of the suspected and high-risk patients of CHD in real-time, from a distant facility.

## Figures and Tables

**Figure 1:** A cardiac cycle of pulse waveform. Notes. The *y*-axis is the amplitude of the pulse signal whose unit is millimeter (mm). The *x-*axis is the time whose unit is second (s).

**Figure 2:** Signal coarse-grained procedure.

**Table 1:** Physiological significances of time-domain features of pulse wave.

No.	Parameters	Physiological significance
1	H2/H1	It reflects the compliance and peripheral resistance of the vascular wall.
2	H3/H1	It reflects the compliance and peripheral resistance of the vascular wall.
3	H4/H1	It reflects peripheral resistance.
4	H5/H1	It reflects the compliance of the aorta and the function of the aortic valve.
5	T(s)	It reflects the pulse wave period.
6	W1(s)	It reflects the duration of high arterial pressure.
7	W2(s)	The duration of maintaining high intravascular pressure.
8	T1/T	It reflects the ejection function of the heart.
9	T1/T4	It reflects the rapid ejection of the heart.

The article "Identifying Coronary Artery Lesions by Feature Analysis of Radial Pulse Wave: A Case-Control Study" was published in 2021. Journal: Biomed Res Int.

**Table 2:** Characteristics of the study subjects.

Factors	Group 1 (*n* = 115)	Group 2 (*n* = 277)	Group 3 (*n* = 137)	*x* ^2^/*F*	*P* value
Male, *n* (%)	67 (58.261)	169 (61.011)	100 (72.993)	7.430	0.024
Female, *n* (%)	48 (41.739)	108 (38.989)	37 (27.00)		
Age (years)	62.98 ± 11.372	66.56 ± 9.779^▲^	66.79 ± 11.641^▲^	4.798	0.009
BMI (kg/m^2^)	24.922 ± 3.461	24.408 ± 3.520	24.364 ± 3.290	1.063	0.347
SBP (mmHg)	135.65 ± 15.261	131.49 ± 16.008^▲^	134.07 ± 14.780	3.293	0.038
DBP (mmHg)	78.58 ± 8.812	77.23 ± 9.049	77.69 ± 6.809	1.031	0.357
Pulse pressure difference (mmHg)	57.07 ± 12.634	54.26 ± 12.428	56.38 ± 13.536	2.490	0.084
History of smoking, *n* (%)	25 (21.740)	73 (26.354)	43 (31.387)	3.003	0.223
History of drinking, *n* (%)	24 (21.739)	33 (11.913)	20 (14.599)	5.241	0.073
Hypertension, *n* (%)	70 (60.870)	186 (67.148)	109 (79.562)	11.143	0.004
Type 2 diabetes, *n* (%)	19 (16.522)	84 (30.324)	72 (52.555)	38.664	0.001
Dyslipidemia, *n* (%)	45 (39.130)	112 (40.433)	70 (51.095)	5.111	0.078
Family history of cardiovascular diseases, *n* (%)	30 (26.087)	46 (16.606)	21 (15.328)	5.995	0.0499
Lack of exercise, *n* (%)	86 (74.783)	227 (81.949)	119 (86.861)	6.123	0.047

Abbreviation: BMI: body mass index; SBP: systolic pressure; DBP: diastolic pressure; definition: history of smoking was defined as subjects who smoked one cigarette or more per day for over 6 months; history of drinking was defined as involving drinking for more than six months and drinking more than 10 grams a day; hypertension was defined as systolic blood pressure ≥ 140 mmHg or diastolic blood pressure ≥ 90 mmHg; type 2 diabetes was defined as fasting blood glucose ≥ 7 mmol/L or postprandial blood sugar ≥ 11 mmol/L; dyslipidemia was defined as total cholesterol ≥ 200 mg/dL, or low-density lipoprotein cholesterol ≥ 130 mg/dL, or high-density lipoprotein cholesterol < 40 mg/dL, or triglyceride ≥ 150 mg/dL; lack of exercise was defined as exercise less than three times a week, and each time less than half an hour; ^▲^compared with Group 1, *P* < 0.05; ^∗^compared with Group 2, *P* < 0.05.

**Table 3:** Comparison of time-domain features between groups with different numbers of coronary artery lesions.

Time-domain features	Group 1 (*n* = 115)	Group 2 (*n* = 277)	Group 3 (*n* = 137)	*Z*	*P* values
H2/H1	0.881 (0.686, 0.954)	0.939 (0.846, 0.973)^▲^	0.927 (0.742, 0.972)	11.690	0.002
H3/H1	0.753 (0.537, 0.842)	0.817 (0.718, 0.893)^▲^	0.776 (0.609, 0.887)	12.448	0.002
T1/T	0.164 (0.130, 0.197)	0.156 (0.123, 0.192)	0.169 (0.141, 0.205)^∗^	7.925	0.019
T	0.824 (0.721, 0.925)	0.851 (0.762, 0.945)	0.817 (0.731, 0.889)^∗^	9.059	0.011
W1	0.199 (0.152, 0.228)	0.211 (0.171, 0.238)	0.194 (0.163, 0.227)^∗^	8.696	0.013
W2	0.148 (0.110, 0.174)	0.164 (0.122, 0.194)^▲^	0.143 (0.118, 0.183)	9.456	0.009

Data shown are M (Q1, Q3); ^▲^compared with Group 1, *P* < 0.05; ^∗^compared with Group 2, *P* < 0.05.

The article "Identifying Coronary Artery Lesions by Feature Analysis of Radial Pulse Wave: A Case-Control Study" was published in 2021. Journal: Biomed Res Int.

**Table 4:** Comparison of multiscale entropy features between groups with different numbers of coronary artery lesions.

MSE	Group 1 (*n* = 115)	Group 2 (*n* = 277)	Group 3 (*n* = 137)	*Z*	*P* value
MSE1	0.045 (0.034, 0.08)	0.040 (0.032, 0.07)	0.039 (0.032, 0.049)^▲^	7.524	0.023
MSE2	0.093 (0.070, 0.168)	0.082 (0.065, 0.145)	0.079 (0.065, 0.101)^▲^	7.535	0.023
MSE3	0.143 (0.107, 0.264)	0.125 (0.099, 0.227)	0.121 (0.100, 0.156)^▲^	7.516	0.023
MSE4	0.194 (0.145, 0.369)	0.171 (0.134, 0.315)	0.164 (0.135, 0.214)^▲^	7.504	0.023
MSE5	0.248 (0.184, 0.484)	0.216 (0.170, 0.411)	0.208 (0.171, 0.272)^▲^	7.344	0.025

^▲^compared with Group 1, *P* < 0.05; ^∗^compared with Group 2, *P* < 0.05.

**Table 5:** Average precisions of stratification models (%).

Classifier	Datasets	Group 1 (*n* = 115)	Group 2 (*n* = 277)	Group 3 (*n* = 137)	Average precision
KNN	Dataset 1	64.24	38.64	65.35	56.07
	Dataset 2	67.51	40.42	61.34	56.44
	Dataset 3	64.25	42.98	64.30	57.17
DT	Dataset 1	75.11	44.06	67.51	62.21
	Dataset 2	76.14	49.45	77.96	67.87
	Dataset 3	78.65	50.50	76.18	68.45
RF	Dataset 1	86.95	55.23	80.51	74.25
	Dataset 2	87.38	72.21	80.86	80.15
	Dataset 3	89.16	67.10	86.65	80.98

## Data Availability

The datasets generated and analyzed during the current study are not publicly available due to the confidentiality of the data, which is an important component of the National Science Foundation of China (No. 82074332) in China, but are available from the corresponding author on reasonable request.

## Abbreviations

CVD: Cardiovascular diseases
CHD: Coronary heart disease
KNN: *k*-nearest neighbors
DT: Decision tree
RF: Random forest
BMI: Body mass index
SBP: Systolic pressure
DBP: Diastolic pressure.
